RETRACTED

# Long non-coding RNA LINC00346 contributes to cisplatin resistance in nasopharyngeal carcinoma by repressing miR-342-5p

**DOI:** 10.1098/rsob.190286

**Published:** 2020-05-13

**Authors:** Zheqing Cui, Tian Pu, Yujie Zhang, Jia Wang, Yulin Zhao

**Affiliations:** 1 Department of Rhinology, the First Affiliated Hospital of Zhengzhou University, No. 1 Jianshe East Road, Zhengzhou, Henan 450052, People's Republic of China; 2 Department of Gastroenterology, the First Affiliated Hospital of Zhengzhou University, No. 1 Jianshe East Road, Zhengzhou, Henan 450052, People's Republic of China

**Keywords:** LINC00346, miR-342-5p, nasopharyngeal carcinoma, cisplatin resistance, lncRNA

## Abstract

Cisplatin has been used as the first-line chemotherapy to treat advanced nasopharyngeal carcinoma (NPC), while acquired cisplatin resistance resulting from epigenetic regulation is not well understood. The relative expression of LINC00346 was detected in healthy persons, cisplatin-sensitive (CS) patients and cisplatin-resistant (CR) patients. The regulatory effect of LINC00346 on the proliferation was detected by cell-counting kit-8. Apoptosis was assayed by histone/DNA ELISA and Caspase-3 activity. Clonal formation and cisplatin resistance were also deciphered. Luciferase reporter and RNA immunoprecipitation assay were adopted to study the interaction between LINC00346 and miR-342-5p. LINC00346 was highly expressed in NPC patients, especially in CR patients, which was associated with cisplatin resistance and poor prognosis. Inhibition of LINC00346 expression promoted cisplatin sensitivity of NPC cells, while LINC00346 over-expression promoted cisplatin resistance of NPC cells. miR-342-5p expression was negatively correlated with cisplatin resistance, and microRNA-342-5p siRNAs treatment could rescue the cisplatin resistance diminished by LINC00346 inhibition. It was further found that miR-342-5p was negatively regulated by LINC00346. In conclusion, LINC00346 regulates the cisplatin resistance of NPC cells by inhibiting miR-342-5p, which could provide a potential target for chemotherapy resistance.

## 1. Introduction

As the most common cancer originating from the nasopharyngeal mucosal lining, nasopharyngeal carcinoma (NPC) commonly affects the postero-lateral nasopharynx or pharyngeal recess, with a relatively higher incidence in East Asia and Africa than elsewhere. Epstein–Barr virus, smoking, diet habits and genetic susceptibility can contribute to the development and pathology of NPC in both children and adults [1–3]. It is worth noting that NPC accounts for about one-third of all upper airway cancers in children. Due to extensive local spread, NPC is usually considered unresettable, and surgery may have a limited treatment effect.

RETRACTED

High-dose radiation therapy alone has a role in the management of NPC. However, clinical practice in both adults and children shows that combined-modality treatment with external beam radiation and cisplatin (also known as DDP)-based chemotherapy is the most effective way to treat NPC, with a cure rate of 70% [1,4,5]. However, about 30% of patients with metastasis will usually develop resistance after six courses of cisplatin chemotherapy [6–8].

Although multiple factors are known to contribute to cisplatin resistance, the detailed molecular regulatory mechanisms related to non-protein coding RNA (ncRNA) have not been fully understood yet. Long intergenic non-protein coding RNA 346 (LINC00346) was shown in previous research to function as an oncogene in gastric cancer, pancreatic cancer and bladder cancer [9–11], which may also play a crucial oncogenic role in NPC and contribute to the development of cisplatin resistance. Cisplatin-resistant NPC cells (CNE1/DDP and CNE2/DDP cells) are constructed in the present study to further decipher the molecular mechanism relevant to LINC00346.

## 2. Methods and materials

### 2.1. Tissue samples

NPC specimens (cisplatin-sensitive, CS; cisplatin-resistant, CR) and adjacent specimens were retrieved from the First Affiliated Hospital of Zhengzhou University. The whole investigation was approved by the Ethics Committee of the First Affiliated Hospital of Zhengzhou University, and written consents were provided by all 50 patients (28 CS and 22 CR).

### 2.2. Cell culture and transfection

Four NPC cell lines (SUNE1, CNE2, HNE1 and C666) and an immortalized nasopharyngeal epithelial cell line (NP69) were ordered from American Type Culture Collection (ATCC). All cell lines were cultured in RPMI-1640 medium (Invitrogen, Carlsbad, CA, USA) supplemented with 10% fetal bovine serum, penicillin (100 U ml^−1^) and streptomycin (100 U ml^−1^), and maintained in a humidified 5% CO_2_ incubator at 37°C. The cisplatin-resistant NPC cells (HNE1/DDP and CNE2/DDP) were established as previously reported [12]. Briefly, parental cell lines CNE1 and CNE2 were cultured with gradually increasing concentrations of cisplatin for six months. The initial concentration of cisplatin was 0.02 µg ml^−1^ and the final concentration was 1 µg ml^−1^. Cisplatin resistance was confirmed by the *in vitro* toxicity test.

### 2.3. Cisplatin sensitivity assay

HNE1/DDP and CNE2/DDP cells were plated into 96-well plates and treated with cisplatin (0.625, 1.25, 2.5, 5.0, 10 and 20 µM) for 48 h. Then, Cell-Counting Kit-8 (CCK-8, Dojindo Laboratories, Tokyo, Japan) was adopted to determine the number of viable cells, and the half-maximal inhibitory concentration (IC_50_) was calculated.

RETRACTED

Caspase-3 Fluorometric Kit (BioVision, Milpitas, CA, USA) and Cell Death Detection ELISAPLUS Kit (Roche Diagnostics, Indianapolis, USA) were used according to the manufacturer's protocol to detect apoptosis.

### 2.4. Colony formation assay

Transfected or untransfected HNE1/DDP and CNE2/DDP cells (1 × 10^3^) were cultured in a six-well plate for two weeks, which was fixed with 4% paraformaldehyde and stained with crystal violet to count the number of colonies.

### 2.5. Small interfering RNAs (siRNAs), plasmids and transfection

LINC00346 small interfering RNAs (siRNAs) (si-LINC00346-1, CAGAACUCAGUUGUCUCUGUAGAAA; si-LINC00346-2, CACAAGGUGUUUGUCCAUCAGUGAU; si-NC, UUCUCCGAACGUGUCACGUdTdT) and miR-342-5p siRNAs were chemically synthesized (Invitrogen, Waltham, MA, USA). For LINC00346 over-expression studies, the whole sequence of LINC00346 (NR_027701.1) was amplified with the following primers (F: AATTA GAATTC AAACGCCCTCCAGGGTG, R: AATTA GGATCC GAAATTTAGCAATTTTCAGAGT), which was further cloned into pcDNA3.1-GFP vector (Invitrogen), named as LINC00346-OE.

### 2.6. Biotin RNA pulldown assay

Sense or antisense biotin-labelled DNA oligomers corresponding to LINC00346 and miR-342-5p (1 μg) were incubated with nuclear extracts from HNE1/DDP and CNE2/DDP cells (2 × 10^7^) for 1 h, then the LINC00346-microRNA complex was isolated with streptavidin-coupled agarose beads (Invitrogen).

### 2.7. Quantitative real-time PCR (qRT-PCR)

RNA (1 µg) extracted from cultured cells or isolated with biotin RNA pulldown method was reverse-transcribed with a High Capacity cDNA Reverse Transcription Kit (Applied Biosystems, Foster City, CA, USA). SYBR Green master mix (Roche, Mannheim, Germany) was used to detect the relative expression and enrichment of LINC00346 and miR-342-5p. The reaction procedures were as follows: 95°C for 10 min, 40 cycles of 95°C for 15 s, and 60°C for 1 min. Expression data were normalized to GAPDH expression. Primer sequences were listed as followed: LINC00346, forward primer 5′-GGAAACGGTCTAGTGGTGGA-3′, reverse primer 5′-AAGCCCTTCTTCACCCTCTC-3′; miR-342-5p, forward primer 5′-ACT AGGGGTGCTATCTGTGA-3′, reverse primer 5′-GTGCAGGGTCCGAGGT-3′; U6 primer, forward primer 5′-CTCGCTTCGGCAGCACA-3′, reverse primer 5′-AACGCTTCACGAATTTGCGT-3′; LINC00346-DNA-1, forward primer 5′-(biotin-) CCTGGACATTCATGGACTTTCGTTTTCACT-3′, reverse primer 5′-(biotin-) AGTGAAAACGAAAGTCCATGAATGTCCAGG-3′; LINC00346-DNA-2, forward primer 5′-(biotin-) TTTCATCCTAAGGAGAAAAAAATGGATTTT-3′, reverse primer 5′-(biotin-) AAAATCCATTTTTTTCTCCTTAGGATGAAA-3′; LINC00346-DNA-3, forward primer 5′-(biotin-) TTTATTGAAAACTGAATATATTAAGATGTG-3′, reverse primer 5′-(biotin-) CACATCTTAATATATTCAGTTTTCAATAAA-3′; GAPDH, forward primer 5′-TATGATGATATCAAGAGGGTAGT-3′, reverse primer 5′-TGTATCCAAACTCATTGTCATAC-3′.

RETRACTED

### 2.8. Luciferase reporter assay

HNE1/DDP and CNE2/DDP cells were first transfected with appropriate miR-342-5p or miR-NC mimics and luciferase reporter vectors containing LINC00346 wild-type (LINC00346-wt) or miR-342-5p-binding-site mutated (LINC00346-mut) segments in 24-well plates for 48 h. Next, HNE1/DDP and CNE2/DDP cells were collected and lysed to detect luciferase activity. The relative luciferase activity was normalized with Renilla luciferase activity.

### 2.9. Statistical analysis

Data were expressed as mean ± standard deviation (s.d.). Both one- and two-way ANOVA with a Tukey's post hoc test, and Student's *t*-test were used. Kaplan−Meier analysis was used to decipher the association between LINC00346 expression and patient survival. At least three independent repeats for the biochemical experiments were conducted for verification of the conclusions. *p* < 0.05 was considered to be statistically significant.

## 3. Results

### 3.1. Upregulated LINC00346 correlates with cisplatin resistance and poor prognosis

The relative expression of LINC00346 was detected in both NPC patients and NPC cell lines with qRT-PCR. LINC00346 expression was remarkably upregulated in primary NPC samples when compared with respective healthy surrounding tissues (figure 1*a*), and a similar upregulated expression trend was also confirmed in the four NPC cell lines (SUNE1, HNE1, C666 and CNE2) and NP69 nasopharyngeal epithelial cell line (figure 1*b*) (*p* < 0.01). It is worth noting that CR patients showed increased LINC00346 expression when compared with CS patients (figure 1*c*). The established cisplatin resistance NPC cells (CNE2/DDP and HNE1/DDP) showed upregulated LINC00346 expression compared with parental NPC cells (HNE1 and CNE2) (figure 1*d*). Kaplan−Meier analysis pointed out that high LINC00346 expression correlated with lower overall survival (figure 1*e*, *p* = 0.0055) and recurrence-free survival (figure 1*f*, *p* = 0.0105) compared with low LINC00346 expression.

**Figure 1.** LINC00346 is upregulated in NPC and associated with cisplatin resistance and poor prognosis. (*a*) The relative expression of LINC00346 in 50 paired NPC specimens and adjacent normal tissues. (*b*) The relative expression of LINC00346 in four human NPC cell lines (SUNE1, HNE1, CNE2 and C666) and NP69, an immortalized nasopharyngeal epithelial cell line. (*c*) The relative expression of LINC00346 in NPC specimens from 28 CS patients and 22 CR patients. (*d*) Relative LINC00346 expression levels of parental NPC cells (HNE1 and CNE2) and cisplatin-resistant NPC cells (HNE1/DDP and CNE2/DDP). (*e,f*) Kaplan−Meier curves in NPC patients with high (*n* = 25) or low LINC00346 expression (*n* = 25) for (*e*) overall and (*f*) recurrence-free survival. **p < 0.01; ***p < 0.001.

RETRACTED

### 3.2. LINC00346 inhibition sensitizes cisplatin-resistant human NPC cells

The biological relevance of LINC00346 in NPC chemosensitivity was deciphered with siRNA transfection and plasmid over-expression method. The success of LINC00346 siRNAs (si-LINC00346-1 and si-LINC00346-2) transfection was confirmed by the detection of diminished LINC00346 expression (figure 2*a*). LINC00346 siRNAs transfection could diminish the tolerance of both HNE1/DDP cells (figure 2*b*) and CNE2/DDP cells (figure 2*c*) to cisplatin as indicated by decreased cell viability. It was further shown that such treatment could inhibit the ability of tumorigenesis suggested by the clonal formation ability of HNE1/DDP cells and CNE2/DDP cells (figure 2*d*). HNE1/DDP and CNE2/DDP cells transfected with LINC00346 siRNAs were treated with different doses of cisplatin for 48 h to determine the IC_50_, which indicated that LINC00346 siRNAs transfection could sensitize NPC cells to cisplatin (figure 2*e*) with increased apoptotic rate determined by Caspase-3 activity assay (figure 2*f*) and histone/DNA ELISA test (figure 2*g*). All of these results indicated that LINC00346 siRNAs transfection could sensitize NPC cells to cisplatin administration by diminished proliferation, tumorigenesis and upregulated apoptosis process.

**Figure 2.** LINC00346 inhibition sensitizes NPC cells to cisplatin. (*a*) Real-time PCR analysis of LINC00346 in CR NPC cells (CNE2/DDP and HNE1/DDP) transfected with LINC00346 siRNAs (si-LINC00346-1, si-LINC00346-2) or negative control siRNA (si-NC). (*b,c*) HNE1/DDP and CNE2/DDP cells transfected with LINC00346 siRNAs or si-NC were treated with different doses of cisplatin for 48 h and analysed with CCK-8 assay. (*d*) Colony formation assay of HNE1/DDP and CNE2/DDP cells treated with 1 µM cisplatin and transfected with LINC00346 siRNAs or si-NC. (*e*) HNE1/DDP and CNE2/DDP cells transfected with LINC00346 siRNAs or si-NC were treated with various concentrations of cisplatin for 48 h to determine the IC_50_ of cisplatin. (*f,g*) Apoptotic rate of HNE1/DDP and CNE2/DDP cells transfected with LINC00346 siRNAs or si-NC with the cisplatin treatment (1 µM) was measured by Caspase-3 activity assay and histone/DNA ELISA. The data show the mean ± s.d. **p < 0.01; ***p < 0.001.

### 3.3. LINC00346 over-expressed NPC cells acquire cisplatin resistance

In addition to the siRNA inhibition assay, the LINC00346 plasmid (LINC00346-OE) was transfected into HNE1 and CNE2 cells to further evaluate the role of LINC00346 in cisplatin sensitivity (figure 3*a*). CCK-8 assay revealed that LINC00346 over-expression could promote the tolerance of both HNE1 (figure 3*b*) and CNE2 (figure 3*c*) cells to cisplatin with increased IC_50_ (figure 3*d*). It was further shown that LINC00346 over-expression could promote the clonal formation ability of both HNE1 and CNE2 cells (figure 3*e*) with a decreased ratio of apoptosis estimated by Caspase-3 activity (figure 3*f*) and histone/DNA ELISA assay (figure 3*g*). All of these data suggested that LINC00346 was vital in cisplatin sensitivity.

RETRACTED

**Figure 3.** Over-expression of LINC00346 promotes cisplatin resistance of NPC cells. (*a*) The relative expression of LINC00346 in HNE1 and CNE2 cells transfected with LINC00346 over-expression plasmid (LINC00346-OE) or empty vector plasmid (VEC). (*b* and *c*) HNE1 and CNE2 cells transfected LINC00346-OE or VEC were treated with different concentrations of cisplatin for 48 h and analysed by CCK-8 assay. (*d*) Colony formation assay of HNE1 and CNE2 cells transfected with LINC00346-OE or VEC. (*e*) HNE1 and CNE2 cells transfected with LINC00346-OE or VEC were treated with cisplatin for 48 h to determine the IC_50_ of cisplatin. (*f,g*) Apoptotic rate of HNE1 and CNE2 cells transfected with LINC00346-OE or VEC with the cisplatin treatment (10 µM) was measured by Caspase-3 activity assay and histone/DNA ELISA. The data show the mean ± s.d. *p < 0.05; **p < 0.01; ***p < 0.001.

### 3.4. LINC00346 negatively regulates miR-342-5p in HNE1/DDP and CNE2/DDP cells

The estimated binding site of LINC00346 and miR-342-5p revealed by Targetscan [13,14] and the schematic of constructed luciferase reporter vectors of LINC00346 wild-type (LINC00346-wt) and LINC00346 mutated (LINC00346-mut) are presented in figure 4*a*. Luciferase reporter assay showed that miR-342-5p could restrain the luciferase activity of the reporting vector containing LINC00346 wild-type sequence significantly in both HNE1/DDP (figure 4*b*) and CNE2/DDP cells (figure 4*c*), while no difference was observed in the reporting vector groups containing LINC00346 mutated sequence. Biotin pull-down assay and following qRT-PCR analysis was used to detect the relative enrichment of LINC00346 and miR-342-5p in HNE1/DDP (figure 4*d*) and CNE2/DDP cells (figure 4*e*), which indicated the direct binding of LINC00346 and miR-342-5p in the HNE1/DDP and CNE2/DDP cells. LINC00346 siRNAs or negative control was transfected into HNE1/DDP and CNE2/DDP cells to test the function of LINC00346 on miR-342-5p expression, which showed upregulated miR-342-5p expression (figure 4*f*). It was further shown that LINC00346 over-expression plasmid (LINC00346-OE) transfection could downregulate miR-342-5p expression in HNE1 and CNE2 cells (figure 4*g*). All of this indicated that LINC00346 could sponge miR-342-5p in HNE1/DDP and CNE2/DDP cells.

RETRACTED

**Figure 4.** MiR-342-5p is negatively regulated by LINC00346. (*a*) The predicted binding sites for miR-342-5p on LINC00346 transcript and schematic of luciferase reporter vectors constructed with LINC00346 wild-type (LINC00346-wt) and the miR-342-5p binding-site mutated (LINC00346-mut) sequences. (*b*,*c*) The luciferase activities detected in HNE1/DDP and CNE2/DDP cells co-transfected with luciferase reporters and miR-342-5p mimics. (*d*,*e*) The relative enrichment of LINC00346 and miR-342-5p detected by biotin pull-down assay. (*f*) The real-time PCR analysis of miR-342-5p in HNE1/DDP and CNE2/DDP cells transfected with LINC00346 siRNAs or si-NC. (*g*) The real-time PCR analysis of miR-342-5p in HNE1 and CNE2 cells transfected with LINC00346-OE or VEC. The data show the mean ± s.d. *p < 0.05; **p < 0.01; n.s. = not significant.

### 3.5. MiR-342-5p over-expression impairs cisplatin resistance in NPC cells

The relative miR-342-5p expression was remarkably downregulated in primary CR patients compared with CS patients (figure 5*a*), which was also observed in HNE1/DDP and CNE2/DDP cells (figure 5*b*). In order to test the association between miR-342-5p and cisplatin sensitization, miR-342-5p mimics or miR-NC (negative control miRNA) was transfected into HNE1/DDP and CNE2/DDP cells to set up miR-342-5p over-expression model (figure 6*a*). The over-expressed miR-342-5p could downregulate the proliferation of HNE1/DDP (figure 6*b*) and CNE2/DDP cells (figure 6*c*) with diminished IC_50_ (figure 6*d*), all of which suggested that MiR-342-5p over-expression could impair NPC cell-associated cisplatin resistance. Further study indicated that miR-342-5p over-expression decreased the clonal formation ability of both HNE1/DDP and CNE2/DDP cells (figure 6*e*) accompanied by increased apoptosis induction as indicated by both Caspase-3 activity assay (figure 6*f*) and histone/DNA ELISA assay (figure 6*g*).

**Figure 5.** The expression level of miR-342-5p negatively correlates with cisplatin resistance. (*a*) miR-342-5p expression in NPC specimens from 28 CS patients and 22 cisplatin-resistant (CR) patients. (*b*) Relative miR-342-5p expression in parental NPC cells and cisplatin-resistant NPC cells. **p < 0.01.

**Figure 6.** MiR-342-5p over-expression impairs resistance to cisplatin in NPC cells. (*a*) miR-342-5p expression in cisplatin-resistant NPC cells transfected with miR-342-5p mimics or miR-NC. (*b,c*) The cell viability of HNE1/DDP and CNE2/DDP cells transfected with miR-342-5p mimics or miR-NC. (*d*) Colony formation assay of HNE1/DDP and CNE2/DDP cells transfected with miR-342-5p mimics or miR-NC. (*e*) HNE1/DDP and CNE2/DDP cells transfected with miR-342-5p mimics or miR-NC were treated with various doses of cisplatin for 48 h to determine the IC_50_. (*f,g*) Apoptotic rate of HNE1/DDP and CNE2/DDP cells transfected with miR-342-5p mimics or miR-NC was measured by histone/DNA ELISA and Caspase-3 activity assay. The data show the mean ± s.d. **p < 0.01; ***p < 0.001.

RETRACTED

### 3.6. miR-342-5p siRNAs rescues the effects of LINC00346 siRNAs inhibition on cisplatin resistance of NPC cells

The association of miR-342-5p and LINC00346 mediated cisplatin resistance was further deciphered in si-LINC00346 and miR-342-5p siRNAs co-transfection system (figure 7*a*). si-LINC00346 co-transfected with miR-342-5p siRNAs could rescue the proliferation of HNE1/DDP (figure 7*b*) and CNE2/DDP cells (figure 7*c*) indicated by CCK-8 assay, and rescue the IC_50_ (figure 7*d*) when compared with si-LINC00346 treatment. The fold change of clonal formation can be rescued by miR-342-5p siRNAs and si-LINC00346 co-transfection (figure 7*e*). Caspase-3 activity (figure 7*f*) and histone/DNA ELISA (figure 7*g*) assay indicated that miR-342-5p inhibition rescued the increased cell apoptosis due to inhibition of LINC00346 in HNE1/DDP and CNE2/DDP cells with the cisplatin treatment (1 µM). All of these data indicated that LINC00346 induced cisplatin resistance was mediated by the sponge effect on the expression of miR-342-5p.

**Figure 7.** miR-342-5p knockdown rescues the effect of LINC00346 inhibition on NPC cell cisplatin resistance. (*a*) miR-342-5p expression in HNE1/DDP and CNE2/DDP cells co-transfected with si-LINC00346 and miR-342-5p-inhibitor. (*b,c*) miR-342-5p inhibition rescues the decreased cell viability due to LINC00346 inhibition on HNE1/DDP and CNE2/DDP cells. (*d*) HNE1/DDP and CNE2/DDP cells co-transfected with si-LINC00346 and miR-342-5p-inhibitor were treated with different concentrations of cisplatin for 48 h to determine the IC_50_. (*e*) MiR-342-5p inhibition rescues the decreased ability of colony formation due to inhibition of LINC00346 expression in HNE1/DDP and CNE2/DDP cells treated 1 µM cisplatin. (*f,g*) Histone/DNA ELISA and Caspase-3 activity assay indicated that miR-342-5p inhibition rescues the increased cell apoptosis due to inhibition of LINC00346 in HNE1/DDP and CNE2/DDP cells with the cisplatin treatment (1 µM). The data show mean ± s.d. **p < 0.01; ***p < 0.001.

## 4. Discussion

In our previous work, we have demonstrated that microRNA-342-3p targets FOXQ1 to suppress the aggressive phenotype of nasopharyngeal carcinoma cells [15]. As to miR-342-5p, which shares the same precursor with miR-342-3p, there is little research in nasopharyngeal carcinoma. Increasing evidence has shown that lncRNAs can sponge microRNAs as competing for endogenous RNAs (ceRNAs), which may be involved in tumour evolution and chemotherapy resistance [16–18]. In this research, it is demonstrated that the relative expression of LINC00346 is correlated with the cisplatin resistance in human samples. *In vitro* investigation also indicates that LINC00346 induced cisplatin resistance is mediated by miR-342-5p, whose inhibition could enhance cisplatin-induced decreased proliferation, downregulated clonal formation ability, and increased apoptosis indicated by Caspase-3 activity and histone/DNA ELISA. Furthermore, LINC00346 inhibition could reverse such effects and sensitize NPC cells to cisplatin. To our knowledge, this may be the first report about the ability of LINC00346 to influence the NPC cells' sensitivity to cisplatin.

RETRACTED

LINC00346 is upregulated in breast cancers, gastric cancer, bladder cancer, non-small cell lung cancer and pancreatic cancer, which exerts oncogenic function to promote cancer cell proliferation, migration and invasion [9,11,19,20]. It is also reported that LINC00346 can contribute to pancreatic ductal adenocarcinoma pathogenesis by activating c-Myc, while in gastric cancer, Myc could modulate LINC00346 to promote tumor progression. [9,10]. All of these indicate the complexity of the LINC00346 mediated regulation network. Despite these clinical observations, little is known regarding the function of LINC00346 mediated chemotherapeutic drug resistance.

Dramatic downregulated miR-342 expression is associated with tamoxifen resistance in both MCF-7/HER2*Δ*16 cell and HER2 negative MCF-7 variants, and such association can also be observed in clinical data; that is, reduced miR-342 expression correlates with tamoxifen resistance [21], while over-expressed miR-342-5p could make HER2 positive breast cancer cells more vulnerable to cellular stress [22–24]. In colon cancer cells, miR-342-5p could target the 3′-UTR of N-a-acetyltransferase 10 protein (NAA10) mRNA for degradation to inhibit the tumorigenesis *in vitro* and *in vivo* [25]. Combined with the inhibitory function of microRNA-342-5p observed in this investigation, all of these data indicate that miR-342-5p restoration may represent a potential therapeutic strategy for NPC.

Primary and secondary cisplatin resistance is a significant limitation to clinical application in chemotherapy [26], which may be attributed to the diversity and complex function of LncRNAs. At the present time, several LncRNA-targeting clinical trials have been performed to demonstrate the clinical feasibility [27]. Our investigation suggests that pathogenic LINC00346 may serve as a potential cisplatin resistance biomarker and therapeutic target for NPC, which may help the response prediction and individually tailored therapy.

RETRACTED

This investigation indicates that LINC00346 contributes to NPC cell growth promotion and cisplatin chemoresistance, which may be explained by the antagonization of miR-342-5p. Future studies could test the participation of LINC00346 in cisplatin resistance in an animal model. In summary, LINC00346 can be considered as a potential target to improve chemotherapeutic efficacy for NPC cells.

## Supplementary Material

Reviewer comments

## Data accessibility

Supporting data are available from a publicly available repository (https://doi.org/10.6084/m9.figshare.11948544).
